The article "Mast cells are the main interleukin 17-positive cells in anticitrullinated protein antibody-positive and -negative rheumatoid arthritis and osteoarthritis synovium" was retracted in 2015. Reason: fabricated or falsified data.

# Mast cells are the main interleukin 17-positive cells in anticitrullinated protein antibody-positive and -negative rheumatoid arthritis and osteoarthritis synovium

**DOI:** 10.1186/ar3466

**Published:** 2011-09-20

**Authors:** Jolien Suurmond, Annemarie L Dorjée, Mariëtte R Boon, Edward F Knol, Tom WJ Huizinga, René EM Toes, Annemie JM Schuerwegh

**Affiliations:** 1 Department of Rheumatology, Leiden University Medical Center, PO Box 9600, Albinusdreef 2, C1-R, NL-2300 RC Leiden, The Netherlands; 2 Department of Dermatology/Allergology, University Medical Center Utrecht, Heidelberglaan 100, NL-3584 CX Utrecht, The Netherlands

## Abstract

**Introduction:**

Mast cells have been implicated to play a functional role in arthritis, especially in autoantibody-positive disease. Among the cytokines involved in rheumatoid arthritis (RA), IL-17 is an important inflammatory mediator. Recent data suggest that the synovial mast cell is a main producer of IL-17, although T cells have also been implicated as prominent IL-17 producers as well. We aimed to identify IL-17 expression by mast cells and T cells in synovium of arthritis patients.

**Methods:**

Synovial samples of anticitrullinated protein antibody-positive (ACPA+) and ACPA-negative (ACPA-) RA and osteoarthritis (OA) patients were stained for IL-17 in combination with CD117 (mast cells), CD3 (T cells) and CD68 (macrophages). Concentrations of IL-17 in synovial fluid were determined by ELISA.

**Results:**

The number of IL-17+ cells in synovium was comparable in all groups. Although the vast majority of IL-17+ cells are mast cells, no difference in the percentage of IL-17+ mast cells was observed. Nonetheless, levels of IL-17 in synovial fluid were increased in ACPA+ RA patients compared to ACPA- RA and OA patients.

**Conclusions:**

The synovial mast cell is the main IL-17+ cell in all three arthritis groups analyzed. These data are relevant for studies aimed at blocking IL-17 in the treatment of arthritis.

## Introduction

Rheumatoid arthritis (RA) is an autoimmune disease characterized by chronic inflammation of the synovial lining of the joint. In the majority of patients with established RA, anticitrullinated protein antibodies (ACPAs) can be found [1]. It is currently believed that ACPA+ and ACPA-RA are two different disease entities, each with its own pathogenesis [2].

Several cell types of the immune system play a role in the pathogenesis of RA. The presence of autoantibodies and the linkage of RA to human leukocyte antigen shared epitope alleles in ACPA+ RA indicate that the adaptive immune system plays a prominent role. However, cells of the innate immune system, such as mast cells, have also been implicated in pathogenesis of RA [3]. Indeed, the number of mast cells in synovial tissue is associated with inflammatory mediators such as histamine in synovial fluid [4].

The article "Mast cells are the main interleukin 17-positive cells in anticitrullinated protein antibody-positive and -negative rheumatoid arthritis and osteoarthritis synovium" was retracted in 2015. Reason: fabricated or falsified data.

Among the cytokines that are thought to be involved in RA, IL-17 has recently attracted considerable attention. IL-17 can induce production of other proinflammatory factors such as IL-6, IL-1, TNF and matrix metalloproteinases, leading to inflammation, breakdown of cartilage and bone erosion [5]. IL-17 deficient mice are less prone to develop experimental arthritis and blocking IL-17 can reduce both the onset and progression in these models [6]. In RA, high levels of IL-17 were found in synovial fluid, especially compared to OA patients [7]. The first proof-of-concept trial indicates that neutralization of IL-17 is a potential new target for the treatment of RA [8].

On the basis of the data described above, it is postulated that Th17 cells, through the production of IL-17 and other Th17-associated cytokines, play a prominent role in the inflamed synovium by perpetuating the inflammatory milieu observed in arthritis [6]. Interestingly, a recent study by Hueber *et al*. [9] indicated that the mast cell is the most abundant cell type expressing IL-17 in the synovial tissue of 10 RA patients. However, other studies have shown the presence of IL-17-producing T cells in RA patients [10]. Because previous investigators have reported that ACPA+ and ACPA- RA are distinct disease entities [2], our aim in the present study was to analyze which cell subsets express IL-17 in the synovial tissue of ACPA+ RA, ACPA-RA and OA patients.

## Materials and methods

### Patient samples

Synovial tissues were obtained from established ACPA+ (*n *= 34) and ACPA- (*n *= 25) RA patients who had undergone therapeutic arthroscopic lavage of an inflamed knee and knee or hip replacement surgery. Synovial tissues were obtained from patients with established OA (*n *= 29) who had undergone knee or hip replacement surgery. These tissues were fixed with 4% formaldehyde in PBS, stored in 70% ethanol and embedded in paraffin. Written informed consent was obtained from the patients, and the study was approved by the Leiden University Medical Center human ethics committee.

Synovial fluid was collected from established ACPA+ RA patients (*n *= 30) and ACPA- RA patients (*n *= 29) and from patients with established OA (*n *= 14) and stored at -20°C until analysis. Patient diagnoses of RA or OA were made according to the American College of Rheumatology criteria [11-13].

### Immunohistochemistry

Synovial tissues were treated according to the method described by Schuerwegh *et al*. [14]. Slides were preincubated with 10% blocking buffer (10% normal horse serum/10% normal human serum in PBS) for 20 minutes and stained with polyclonal goat anti-human IL-17A (0.50 μg/mL; R&D Systems, Minneapolis, MN, USA) in 1% blocking buffer (1% normal horse serum/1% normal human serum in PBS/1% BSA) for one hour. For control sections, a matching isotype control (normal goat immunoglobulin G (IgG); Merck, Darmstadt, Germany) was used. Detection was performed using horse α-goat biotin (Vector Laboratories, Burlingame, CA, USA), avidin-biotin-peroxidase complex (VECTASTAIN Elite ABC Kit; Vector Laboratories) and 3, 3'-diaminobenzidine tetrahydrochloride-nickel chloride (Vector Laboratories).

The article "Mast cells are the main interleukin 17-positive cells in anticitrullinated protein antibody-positive and -negative rheumatoid arthritis and osteoarthritis synovium" was retracted in 2015. Reason: fabricated or falsified data.

For combined staining of IL-17 with CD117, CD3, CD4 or CD68, slides were stained for one hour with polyclonal rabbit anti-human CD117 (23 μg/mL; Dako, Glostrup, Denmark), monoclonal mouse anti-human CD3 (2.8 μg/mL; Dako), monoclonal mouse anti-human CD4 (7 μg/mL; Dako), monoclonal mouse anti-human CD68 (0.51 μg/mL; Dako) or matching isotype control (rabbit polyclonal Ig and mouse IgG1; Dako) in 1% blocking buffer. Detection of anti-CD117, anti-CD3, anti-CD4 or anti-CD68 was performed using alkaline phosphatase-conjugated anti-rabbit/anti-mouse Ig and Liquid Permanent Red (EnVision™ G|2 System/AP, Rabbit/Mouse (Permanent Red) Kit; Dako). The tissue sections were counterstained with hematoxylin.

Stained sections were coded and randomly analyzed. The mean number of single- and double-positive cells in 10 high-power fields (original magnification, ×400) was scored blindly by two observers.

### Immunoassay for IL-17

Concentrations of IL-17A in synovial fluid were measured with an ELISA (PeproTech, Inc., Rocky Hill, NJ, USA) according to the manufacturer's instructions.

### Statistical analysis

Differences between patient and control groups were analyzed using the Kruskal-Wallis and Mann-Whitney *U *tests. In all tests, *P *< 0.05 was considered significant.

## Results

To determine the expression of IL-17 by mast cells, T cells and macrophages in synovial tissue, immunohistochemical staining was performed in synovial tissue sections of ACPA+ RA, ACPA- RA and OA patients (Table 1). Representative examples of the staining are shown in Figure 1. Isotype controls were negative (data not shown).

**Table 1:** Expression of IL-17 by mast cells, T cells and macrophages in synovial tissue

Demographics	ACPA+ RA (*n *= 34)	ACPA- RA (*n *= 25)	OA (*n *= 29)	*P *value
Age (years)	55 (32 to 80)	63 (19 to 80)	67 (42 to 83)	
Gender (females/males)	22/12	14/11	21/8	
Disease duration (years)	7 (0 to 28)	8 (0 to 24)	Unknown	
Median IL-17+ cells	21 (0 to 118)	12 (1 to 61)	17 (0 to 50)	0.381
IL-17+ mast cells (%)	97 (40 to 100)	96 (0 to 100)	93 (0 to 100)	0.969
IL-17+ T cells (%)	0 (0 to 100)	0 (0 to 24)	2 (0 to 49)	0.558
IL-17+ MØ (%)	0 (0 to 78)	4 (0 to 100)	1 (0 to 58)	0.382
Median MCs	28 (0 to 123)	19 (0 to 92)	25 (0 to 76)	0.198
MCs (CD117+) expressing IL-17 (%)	91 (13 to 100)	83 (0 to 100)	96 (4 to 100)	0.599
T cells (CD3+), *n*	21 (0 to 592)	10 (0 to 115)	11 (0 to 265)	0.609
T cells (CD3+) expressing IL-17 (%)	0 (0 to 60)	0 (0 to 66)	1 (0 to 78)	0.149
MØ (CD68+), *n*	71 (1 to 390)	53 (1 to 302)	66 (2 to 231)	0.634
MØ (CD68+) expressing IL-17 (%)	0 (0 to 16)	0 (0 to 14)	0 (0 to 11)	0.689

ACPA: anticitrullinated protein antibody; MC: mast cell; MØ: macrophage; OA: osteoarthritis; RA: rheumatoid arthritis. Results are expressed as medians (minimum-maximum). Mast cells are defined as CD117+ cells, T cells are defined as CD3+ cells and macrophages are defined as CD68+ cells.

The article "Mast cells are the main interleukin 17-positive cells in anticitrullinated protein antibody-positive and -negative rheumatoid arthritis and osteoarthritis synovium" was retracted in 2015. Reason: fabricated or falsified data.

**Figure 1:** **Expression of IL-17 by immunohistochemistry**. **(A) **Double-staining of IL-17 (black) and CD117+ mast cells (pink). **(B) **Double-staining of IL-17 (black) and CD68+ macrophages (pink). **(C) **Double-staining of IL-17 (black) and CD3+ T cells (pink). **(D) **Double-staining of IL-17 (black) and CD4 (pink). Representative examples are shown. In insets in parts **(A) **through **(D)**, arrows indicate double-positive cells and arrowheads indicate single IL-17+ cells. The magnification of inset images are made digitally, and are 2× the magnification of the original figure which is made through a 400× magnification.

The median number of IL-17+ cells was slightly higher in ACPA+ RA patients than in ACPA- RA and OA patients, but this difference was not statistically significant (Figure 2A). Likewise, the total number of CD117+ cells was slightly higher in ACPA+ RA patients, although the difference was not statistically significant. There was no difference in the number of T cells (CD3+) or macrophages (CD68+) between the groups.

**Figure 2:** **IL-17 in synovial tissue and synovial fluid**. **(A) **Number of IL-17+ cells in synovial tissue of ACPA- and ACPA+ RA and OA patients. The results are expressed as the number of cells assessed in 10 high-power fields at ×400 magnification. **(B) **Levels of IL-17 in synovial fluid determined by ELISA. *P < 0.05 and **P < 0.01, both indicating statistically significant differences. ACPA, anticitrullinated protein antibody; OA, osteoarthritis; RA, rheumatoid arthritis.

To identify the source of IL-17 in synovium, double-staining of IL-17 with CD117 (mast cells), CD3 (T cells) and CD68 (macrophages) was performed. Interestingly, almost all IL-17-expressing cells were CD117+ in the synovial tissue of ACPA+ and ACPA- RA patients as well as OA patients. Only a small fraction of IL-17+ cells were CD3+ or CD68+ (Table 1). Furthermore, there were no differences in these percentages between the three groups. Because CD3 can be downregulated in activated T cells, we performed additional staining of IL-17 in combination with CD4 in six synovium samples (Figure 1D). The median percentage (minimum-maximum range) percentage of IL-17+ cells that were CD4+ was 0.4% (0.0% to 11.0%). The median (minimum-maximum range) percentage of CD4+ cells that were IL-17+ was 0.1% (0.0% to 0.7%). Taken together, these data indicate that IL-17 in synovium is expressed predominantly by mast cells.

The article "Mast cells are the main interleukin 17-positive cells in anticitrullinated protein antibody-positive and -negative rheumatoid arthritis and osteoarthritis synovium" was retracted in 2015. Reason: fabricated or falsified data.

Since immunohistochemistry does not reveal secretion of IL-17, an ELISA was performed with the synovial fluid of RA and OA patients. ACPA+ RA patients had significantly higher levels of IL-17 in synovial fluid compared to ACPA- RA and OA patients (Figure 2B).

## Discussion

In this study, we have shown in a relatively large group of 59 RA and 29 OA patients that the majority of IL-17+ cells were mast cells and not T cells or macrophages. Interestingly, levels of IL-17 in synovial fluid were increased in ACPA+ RA patients. Because the expression of IL-17 in synovial tissue correlates strongly with the number of mast cells, it is conceivable that the increased level of IL-17 in the synovial fluid of ACPA+ RA patients results from the increased activity of mast cells in ACPA+ RA patients. Our data also show that IL-17 is not increased in all ACPA+ RA patients. Preliminary analysis of the characteristics of the RA patients with a high number of IL-17-producing cells shows that these patients tend to have higher serum ACPA titers and erythrocyte sedimentation rates at the time of diagnosis.

In this study, mast cells were identified as CD117+ cells. As described in Schuerwegh *et al*. [14], flow cytometric staining of synovial tissue revealed that all CD117+ cells express the high-affinity IgE receptor (FcεRI) and/or IgE. Therefore, CD117 alone can be considered a good mast cell marker in synovial tissue.

Although our results suggest that mast cells are the most prominent producers of IL-17 in synovial tissue, a clear limitation of this study is that only the expression of IL-17, and not active secretion, was studied. We do not know whether IL-17 is secreted by activated mast cells, as we were unable to isolate viable mast cells from synovial tissue. Nonetheless, Hueber *et al*. [9] showed IL-17 secretion by *in vitro *cultured mast cells, indicating that mast cells can readily produce IL-17. Because the samples of synovial fluid, in which higher levels of IL-17 were found, were from different patients than the samples of synovial tissue, it is unclear whether the increased levels of IL-17 correlate directly to the presence of IL-17+ mast cells in the same synovial tissue.

The article "Mast cells are the main interleukin 17-positive cells in anticitrullinated protein antibody-positive and -negative rheumatoid arthritis and osteoarthritis synovium" was retracted in 2015. Reason: fabricated or falsified data.

Our group previously found that IgE-ACPA can bind to FcεRI on basophils and that citrullinated proteins can directly activate basophils of ACPA+ RA patients. In addition, an increased number of degranulated mast cells was shown in the synovium of ACPA+ RA patients, indicating a higher activity of mast cells in these patients [14]. Because mast cells also express FcεRI, it is tempting to speculate that mast cells are also activated by citrullinated proteins present in the joint, thereby releasing IL-17, which contributes to the inflammatory milieu present in the inflamed synovium. However, there was no difference in the expression of IL-17 between ACPA+ and ACPA- RA patients in our study. Therefore, it is unclear whether the more activated state of mast cells that was found before [14] is related to the release of IL-17, as in our present study we were able to evaluate only the expression of IL-17 rather than its secretion.

Several studies have provided evidence indicating that IL-17-producing T cells in synovial tissue or fluid also contribute to inflammation. However, these T cells are not abundantly present in the synovial compartment. Indeed, even after strong nonspecific T-cell triggering, only a small minority of CD4+ T cells (about 1% to 10%) obtained from synovial fluid or synovial tissue produce IL-17, as shown by flow cytometry [10,15-17]. Furthermore, the antigen specificity of these Th17 cells in synovium is unknown; therefore, these cells can also be innocent bystanders that do not contribute to inflammation in the joint *in vivo*. In two studies in which immunohistochemical staining was performed, IL-17+ cells were identified as CD3+ cells. However, it is unclear how these results relate to our study, as in those previous studies cells were identified using single staining of consecutive sections and the positive cells in the overlying sections were not quantified, making it difficult to compare these contradictory results with the results of our study [18,19]. Two other studies in which microscopic analysis was performed showed that almost no CD3+ T cells in the synovium expressed IL-17. In agreement with our study, in one of these studies the cell types that did express IL-17 were found to be mainly mast cells [9]. However, the other study in which no CD3+ T cells were shown to express IL-17 identified IL-17+ cells as being mainly neutrophils and neutrophil precursors in the synovium of the facet joints [20]. Because we found the mast cells to be the main cell subset expressing IL-17 in synovium from the knee, it is possible that the cells expressing IL-17 might be different, depending on the site of the joint.

The article "Mast cells are the main interleukin 17-positive cells in anticitrullinated protein antibody-positive and -negative rheumatoid arthritis and osteoarthritis synovium" was retracted in 2015. Reason: fabricated or falsified data.

Because the production of IL-17 is highly restricted by transcriptional control via RORγT (retinoid acid receptor-related orphan receptor γt), which is also known to regulate the production of other Th17-associated cytokines, mast cells might also produce other Th17-related cytokines, such as IL-22. Furthermore, because mast cells can produce many other cytokines as well, blocking the activation of mast cells, such as by preventing their activation via the FcεRI through anti-IgE treatment, might lead to even more profound effects than blocking IL-17 alone in arthritis patients. Indeed, blocking TNF is a very successful therapy in RA, and mast cells are known to be important producers of TNF [21].

## Conclusions

Our results show that IL-17 is expressed mainly by mast cells in the synovial tissue of both ACPA+ and ACPA- RA patients, as well as in OA patients. Selective activation of mast cells in ACPA+ RA patients might be responsible for the increased levels of IL-17 in synovial fluid. These data are relevant for new targeted therapies in arthritis, such as IL-17 blockade or the inhibition of mast cell activation.

## Abbreviations

ACPA: anticitrullinated protein antibodies; BSA: bovine serum albumin; ELISA: enzyme-linked immunosorbent assay; IL: interleukin; OA: osteoarthritis; PBS: phosphate-buffered saline; RA: rheumatoid arthritis; TNF: tumor necrosis factor.

## Competing interests

The authors declare that they have no competing interests.

## Authors' contributions

JS carried out the experiments, performed the statistical analysis and drafted the manuscript. AD and MB carried out the experiments and contributed to the design and analysis of the study. EK, TH, RT and AS participated in the design and analysis of the study and helped to draft the manuscript. All authors read and approved the final manuscript.
